This article has been retracted.

# NDRG4 Alleviates Myocardial Infarction-Induced Apoptosis through the JAK2/STAT3 Pathway

**DOI:** 10.1155/2022/4869470

**Published:** 2022-01-27

**Authors:** Changliang Zhao, Yuanyuan Ren, Yachao Zhang

**Affiliations:** ^1^Department of Cardiology 4, The Third Affiliated Hospital of Qiqihar Medical University, Qiqihar, 161000 Heilongjiang, China; ^2^Intensive Care Unit, Hospital of Traditional Chinese Medicine of Qiqihar, Qiqihar, 161000 Heilongjiang, China

## Abstract

**Objective:**

At present, studies have confirmed that NDRG4 is specifically expressed in the heart, while its effect on the heart is still unclear. This study is to explore the effect of NDRG4 on cardiomyocyte apoptosis caused by acute myocardial infarction (AMI).

**Methods:**

Twenty SD rats were randomly divided into Sham (left anterior descent of heart without ligation) and AMI groups. In this study, coronary artery ligation was used to establish an AMI model, and the AMI model was verified by auxiliary examination and pathological examination. Besides, quantitative real-time polymerase chain reaction (qRT-PCR) and Western blotting (WB) was used to detect the expression level of Bax and Bcl-2 in heart tissues, and NDRG mRNA levels in tissues were also detected. qRT-PCR technology was used to verify the transfection efficiency of NDRG4 in H9C2 cells, and the change of apoptosis level of H9C2 cells was detected by Cell Counting Kit-8 (CCK-8) assay and TUNEL staining; besides, the expression level of apoptosis-related factors was detected by WB and qRT-PCR technology. Simultaneously with the modeling of rats, we injected adenovirus (Ad) into the heart tissue and examined the structural and functional changes of the rat heart. Then, WB technology was used to detect the expression level of the JAK2/STAT3 signaling pathway.

**Results:**

The heart function and heart structure of rats in the MI group were dramatically worse, and the expression level of NDRG4 was also dramatically reduced. The overexpression of NDRG4 in H9C2 cells can effectively inhibit the ischemia/hypoxia- (I/H-) induced decrease in cell viability and increase in apoptosis rate and inhibit the increase in Bax/Bcl-2 ratio. Moreover, overexpression of NDRG4 in heart tissue can effectively improve the cardiac function and structural destruction caused by MI. In addition, NDRG4 can inhibit JAK2/STAT3 pathway activation.

**Conclusion:**

The expression of NDRG4 in the MI tissue of rats was suppressed, while overexpression of NDRG4 by injection of Ad can obviously protect the rat heart. Furthermore, overexpression of NDRG4 in H9C2 cells can effectively inhibit the I/H-induced decrease in cell viability and increase in apoptosis rate, and this may be related to the inhibition of the JAK2/STAT3 signaling pathway.

## 1. Introduction

With the increasing prevalence of cardiovascular disease (CVD), it has replaced infectious diseases as the “number one killer” threatening the health and life of all human beings; the most common of which include ischemic cardiomyopathy (IHD), hypertension, and arrhythmia [1]. IHD with cardiomyocyte death as the basic pathological change is a CVD with high morbidity and mortality worldwide [2, 3]. The methods of cell death after MI are mainly divided into apoptosis and necrosis, and cell apoptosis plays a crucial role in the occurrence and development of heart failure (HF) after MI [2]. Myocardial cells undergo apoptosis, induce inflammation, and stimulate fibrocyte proliferation, which affects cardiac function of patients to a great extent. Moreover, as myocardial cells are terminally differentiated cells and lose regeneration ability, when the apoptosis is too severe, the recovery of cardiac function will be affected to a great extent. Therefore, early regulation of myocardial cell apoptosis is of great significance for the recovery of cardiac function [3]. In our country, AMI is still one of the main causes of death in patients with CVD, and the prognosis of patients depends on the degree of cardiomyocyte apoptosis after MI [4].

N-myc downstream regulatory gene (NDRG) family protein members include NDRG1, NDRG2, NDRG3, and NDRG4, which are composed of about 340-394 amino acid residues and share a common gene sequence of about 53-65% [5]. A large number of studies have confirmed that NDRG family protein members play a crucial role in growth and development, cell proliferation, stress response, endocrine regulation, tumor gene regulation, and apoptosis [6–8]. Moreover, recent studies have found that NDRG4 is also expressed in cardiomyocytes [9]. Therefore, we speculate that NDRG4 also plays an indispensable role in the process of AMI and may be helpful in the prognosis of MI.

Janus kinase/signal transduction and activator of transcription (JAK/STAT) pathways are important intracellular signal transduction pathways that have received much attention in recent years and are involved in mediating many physiological processes such as cell growth, proliferation and differentiation, inflammation, and apoptosis [10–12]. Under physiological conditions, JAK is mainly distributed in the cytoplasm and is in a static or weakly activated state. When cells are properly stimulated, they are rapidly phosphorylated and activated, and the activated JAK/STAT pathway mediates the biological activity of downstream substrate molecules through phosphorylation. In recent years, the role of the JAK2/STAT3 pathway in the pathogenesis of heart disease has attracted much attention. Cardiac hypertrophy, HF, myocardial protection induced by ischemic preconditioning, and cardiac dysfunction induced by ischemia-reperfusion (I/R) are all closely related to this relatively simple signaling pathway [13, 14]. Therefore, we speculated that the JAK2/STAT3 pathway is closely related to AMI and cardiomyocyte apoptosis.

## 2. Materials and Method

### 2.1. Animals and Models

SD rats were anesthetized with 1% pentobarbital sodium (50 mg/kg) by intraperitoneal injection. After tracheal intubation in rats, small animal ventilator was used to assist breathing. Next, the 4th or 5th intercostal muscles were separated and the thoracic cavity was opened; the anterior descending branch of the left coronary artery was ligated at a distance of about 3 mm from the left atrial appendage to the root of the aorta at the conical distance of the pulmonary artery. The Sham group rats' chest was opened and the pericardium cut, while the thread was not ligated at the corresponding part. ST segment elevation of more than 1/2 and paleness of the front wall of the left ventricle on electrocardiogram were considered as the success of the AMI model [15]. At the same time, the NDRG4-overexpressing Ad constructed by Ki Gen Company was used for intramyocardial injection. Simultaneously with rat modeling, a microinjection needle was used to inject 10 *μ*L of Ad into the left ventricle of each rat. The chest was sutured layer by layer, and tracheal intubation was removed after recovery of spontaneous breathing. This experiment has been approved by the Animal Ethics Committee of Qiqihar Medical University (IACUC-1709019).

### 2.2. Rat Hemodynamics and Echocardiography

Transthoracic echocardiography (Visual Sonics, Toronto, Canada) was used to measure the left ventricular end-systolic diameter (LVESD), left ventricular end-diastolic diameter (LVEDD), interventricular septal thickness at diastole (IVSD), left ventricular posterior wall thickness (LVPWT), left ventricular shortening fraction (FS%), and left ventricular ejection fraction (EF%). Biological function collection system BL-420S (Techman, Chengdu, China) was used to detect left ventricular end diastolic pressure (LVEDP), left ventricular developed pressure (LVDP), and left ventricular pressure maximum rise and decline rate (±dp/dt).

### 2.3. Hematoxylin-Eosin Staining

The heart of the rat was taken and immersed in 10% formaldehyde solution for fixation. The tissue was prepared by paraffin infiltration and paraffin embedding to prepare paraffin sections. Then, the sections were placed under an optical microscope (Olympus, Japan) to observe the pathological changes of heart tissue.

### 2.4. Immunohistochemical Staining

Heart tissue sections were dewaxed and dehydrated separately, and 3% H_2_O_2_ was used to block the endogenous peroxidase. Subsequently, 0.5% BSA was blocked by incubation at 37°C for 30 minutes. The primary antibody (Caspase3, Abcam, Cambridge, MA, USA, Rabbit, 1 : 1000) was incubated overnight at 4°C. The next day, the sections were taken to room temperature and left for 30 minutes, and the secondary antibody was added dropwise and incubated at 37°C for 1 hour. Diaminobenzidine (DAB; Yifei Xue, Nanjing, China) was used for tissue color development. After hematoxylin counterstaining, neutral gum was used for sealing. The sections were placed under an optical microscope to observe the positive points.

### 2.5. Cell Culture

H9C2 cardiomyocytes were purchased from the American Type Culture Collection (ATCC, Manassas, Virginia), and the cells were cultured in a Dulbecco's modification of Eagle's medium Dulbecco medium (DMEM; Gibco, Grand Island, NY, USA) containing 10% Fetal Bovine Serum (FBS; Gibco, Grand Island, NY, USA) and supplemented with 1% penicillin and 1% streptomycin in a constant temperature incubator at 37°C and 5% CO_2_ to cultivate. It was used for subsequent experiments when the cells were in the logarithmic growth phase.

### 2.6. Cell Transfection

NDRG4 overexpression plasmid was constructed and transfected when the cell density reached 60%-70%. 125 *μ*L Opti-MEM medium (Gene, Shanghai, China) and 5 *μ*L Lipofectamine^3000^ Reagent (Gene, Shanghai, China) were added in tube A. 125 *μ*L Opti-MEM medium, 5 *μ*L Lipofectamine^3000^ Reagent, and 1 *μ*g plasmid (Gene, Shanghai, China) were added in tube B. Then, mix tubes A and B and let it stand for 5 minutes. The mixed solution was added to the cell culture dish. After 24 hours of transfection, the intervention was performed [16].

### 2.7. Establishment of an I/H Model of H9C2 Cell

When H9C2 cells grow above 80% confluence, the original culture medium was discarded, replaced with serum-free medium, and cells were further cultured in a culture environment of 10% CO_2_ and 1% O_2_. All cells were divided into 4 groups: (1) Normoxia group: normal culture of H9C2 cells; (2) I/H group: H9C2 cells were cultured in an anoxic environment and serum-free medium; (3) I/H+OE-NDRG4 group: H9C2 cells transfected with NDRG4 by plasmid were cultured in an anoxic environment and serum-free medium; (4) I/H+OE-NC group: H9C2 cells transfected with NC by plasmid were cultured in an anoxic environment and serum-free medium.

### 2.8. Cell Counting Kit-8 Assay

After cell treatment, 10 *μ*L of CCK-8 solution (Construction, Nanjing, China) was added to each well, and the incubation was continued in the incubator. After 2 hours, the culture was terminated. Finally, the microplate reader was used to measure OV450 value, and the cell survival rate was calculated according to the formula.

### 2.9. Western Blot

Cells and tissue proteins were extracted with 500 *μ*L of prechilled RIPA protein lysis buffer (Thermo Fisher Scientific, Waltham, MA, USA). After centrifugation at 4°C and 12,000 r/min for 15 minutes, the bicinchoninic acid (BCA; Beyotime, Nanjing, China) was used to determine the protein concentration of the supernatant. 30 *μ*g per well of cell lysed protein was loaded and separated by sodium dodecyl sulfate-polyacrylamide gel electrophoresis (SDS-PAGE). The protein was transferred to the polyvinylidene difluoride (PVDF, Thermo Fisher Scientific, Waltham, MA, USA) membrane. The 5% skim milk powder was incubated with the PVDF membrane at 37°C for 1 hour. Then, the antibodies were added at 4°C overnight. After washing the membrane, horseradish peroxidase-labeled goat anti-mouse or goat anti-rabbit second antibody was added and incubated at 37°C for 1 hour. After washing the membrane, prolight HRP chemiluminescence reagent was added, developed by Odyssey Fc imaging system, and Western blot bands were quantitatively analyzed with ImageJ analysis software. Antibodies are shown in Table S1.

### 2.10. Quantitative Real-Time Polymerase Chain Reaction

TRIzol reagent (Thermo Fisher Scientific, Waltham, MA, USA) was used to extract total RNA from tissues and cells and then reversed transcribed into cDNA according to kit steps. Real-time quantitative PCR uses a 20 *μ*L reaction system: SYBR Premix Ex Taq II 10 *μ*L, ROX Reference Dye 0.4 *μ*L, cDNA 2 *μ*L, forward and reverse primers each 0.8 *μ*L, and RNA-free water 0.6 *μ*L. The reaction conditions are as follows: 95°C 30 s; 95°C 5 s, 55°C 30 s, and 72°C 30 s, a total of 40 cycles. The Ct values of the three replicate wells were used as the average, and the relative fold change in mRNA expression was calculated using the formula 2^-△△CT^. Primers are shown in Table S2.

### 2.11. Enzyme-Linked Immunosorbent Assay (Elisa)

50 *μ*L cell supernatant or rat serum was added to an Elisa plate, and then, 100 *μ*L of horseradish peroxidase detection antibody (LDH or CK-MB) was added to each well and incubated at 37°C for 1 hour. Then, the liquid in the wells was discarded, phosphate-buffered saline (PBS) was used to wash three times, and then, 50 *μ*L of substrates A and B (BD Pharmingen, Shanghai, China) was added to each well and incubated at 37°C in the dark for 15 minutes. Finally, 50 *μ*L of stop solution was added to each well, and the OD value of each well was measured at the wavelength of 450 nm.

### 2.12. TUNEL Staining

The cell intervention of each group in the 24-well plate was as described above, without culture medium, and washed once with PBS. Cells were fixed with immunostaining fixative solution for 1 hour and washed once with PBS. Then, 50 *μ*L TUNEL detection solution (BD Pharmingen, Shanghai, China) was added dropwise to each well and incubated at 37°C in the dark for 1 hour. After being washed three times with PBS, the culture plate was placed under a fluorescent microscope for observation.

### 2.13. Statistical Analysis

SPSS 21.0 software was used for statistical analysis. The data were expressed as mean ± standard deviation (^−^*X* ± SD), one-way ANOVA was used for comparison between groups, and SNK-q was used for pairwise comparison between groups. The test showed that *P* < 0.05 was considered statistically significant.

## 3. Results

### 3.1. Changes of Cardiac Function and Structure after MI in Rats

First, we used echocardiography to detect the rat's cardiac function and ventricular remodeling in the MI and Sham groups. This study found that compared with those in the Sham group, LVESD, LVEDD, and IVSD of rats in the MI group were dramatically increased, while LVPWT, FS%, and EF% were dramatically decreased. In addition, this study also observed that MI group rats' LVEDP dramatically increased, while the LVDP and ±dp/dt dramatically decreased (Figures 1(a)–1(j)). At the same time, Elisa was used to detect the serum of two groups of rats, and it was found that the activities of LDH and CK-MB in the MI group were dramatically increased (Figures 1(k) and 1(l)). H&E staining results showed that the myocardial fibers in the Sham group were neatly arranged and stained uniformly. In the MI group, the myocardial fiber was broken and disordered, and the myocardial cells in the anterior wall of the left ventricle were extensively necrosis, which involved the whole layer of the ventricular wall (Figure 1(m)).

### 3.2. MI Induces Myocardial Cell Apoptosis and Downregulation of NDRG Expression

In order to further clarify the degree of myocardial cell apoptosis after MI, we found by immunohistochemical staining that Caspase3 expression was dramatically upregulated in the MI group (Figure 2(a)). Next, we used WB technology to detect the expression of apoptosis-related factors Bax, Bcl-XL, and Bcl-2 in myocardial tissue (Figure 2(b)). Compared with the Sham group, Bax expression was dramatically increased in the MI group, while Bcl-XL and Bcl-2 expression was dramatically suppressed. At the same time, qRT-PCR also obtained similar results to the former (Figure 2(c)). Next, we used qRT-PCR technology to detect the mRNA levels of NDRG1, NDRG2, NDRG3, and NDRG4 in the heart tissues of the two groups (Figure 2(d)). The results showed that the expression of the above genes in the MI group was suppressed, and we found that NDRG4 expression was most dramatically inhibited in the MI group. Therefore, we speculated that the function of NDRG4 might be more important in AMI, so we carried out the study of NDRG4 in myocardial cells.

### 3.3. Overexpression of NDRG4 Can Inhibit H9C2 cell Apoptosis Induced by I/H Treatment

Next, we transfected OE-NDRG4 into H9C2 cells to observe the effect of I/H treatment on H9C2 cells. We first detected the expression of NDRG4 by qRT-PCR and determined that it was overexpressed in H9C2 cells (Figure 3(a)). To further examine the protective effect of NDRG4 on H9C2 cells, we observed that compared with the I/H group, the activity of H9C2 cells in the I/H+OE-NDRG4 group was dramatically increased (Figure 3(b)), the content of myocardial injury markers LDH and CK-MB was dramatically reduced (Figures 3(c) and 3(d)), and the rate of apoptosis was also reduced (Figure 3(e)). In addition, WB and qRT-PCR detected the expression of Bax, BCL-XL, and Bcl-2 in the four groups of cells. The results showed that overexpression of NDRG4 in H9C2 cells can effectively inhibit the increase of Bax expression and the decrease of Bcl-XL and Bcl-2 expression induced by I/H treatment (Figures 3(f) and 3(g)).

### 3.4. Overexpression of NDRG4 in Rat Heart Can Improve MI-Induced Cardiac Function and Structural Damage

To clarify the protective role of NDRG4 in cardiac tissue, we injected Ad-NDRG4 into the left ventricle while modeling in rats. After 1 day, the expression level of NDRG4 in heart tissue was detected by qRT-PCR technology. The results showed that the NDRG4 mRNA expression level in the MI+Ad-NDRG4 group was higher than that in the MI group (Figure 4(a)). At the same time, we used echocardiography to detect rat heart function and ventricular remodeling. The results showed that compared with the MI group, the LVESD, LVEDD, and IVSD in the MI+Ad-NDRG4 group were dramatically reduced, and the LVPWT, FS%, and EF% were dramatically increased (Figures 4(b)–4(g)). In addition, this study also observed a significant decrease in LVEDP and a significant increase in LVDP and ±dp/dt in the MI+Ad-NDRG4 group (Figures 4(h)–4(k)). Moreover, Elisa found that CK-MB and LDH activity were dramatically reduced in the MI+Ad-NDRG4 group (Figures 4(l) and 4(m)). Also, H&E staining results showed that compared with the MI group, the myocardial muscle fibers were neatly arranged and the myocardial fiber breakage was dramatically reduced in the MI+Ad-NDGR4 group (Figure 4(n)).

### 3.5. NDRG4 Inhibits the Activation of the JAK2/STAT3 Pathway Induced by I/H Treatment

The study found that the JAK2/STAT3 pathway is lowly activated in normal tissues, and when the tissue is stimulated by certain factors, the JAK2/STAT3 pathway will be activated [17]. Therefore, we continued the study after transfecting H9C2 cells with OE-NDRG4 or OE-NC. The results showed that the expressions of p-JAK2 and p-STAT3 in the I/H group were upregulated, while compared with the I/H group, the expressions of p-JAK2 and p-STAT3 in the I/H+OE-NDRG4 group were dramatically suppressed, and p-JAK2/ JAK2 and p-STAT3/STAT3 ratio was dramatically reduced (Figures 5(a) and 5(b)). From this, we speculated that NDRG4 can negatively regulate the JAK2/STAT3 pathway activation, thereby protecting H9C2 cells.

## 4. Discussion

At present, the morbidity and mortality of CVDs in our country are increasing year by year, and IHD is mainly due to insufficient coronary blood flow caused by various reasons, which is difficult to meet the myocardial damage caused by myocardium to energy [18]. At present, coronary bypass or thrombolysis is mainly used to improve the blood supply of the myocardium and protect the ischemic myocardium, but there are many postoperative complications, which makes the effect not ideal [19, 20]. Therefore, finding new therapeutic targets will provide new theories for clinical treatment. In this study, coronary ligation method was used to build an AMI model. This is the most valuable and easy to promote AMI model production method among various AMI models. And when we removed the rat heart, we can clearly see the left ventricle enlargement, ischemic ventricular wall becomes very weak, epicardial and lining in fibrosis in ischemia area, the ischemia area room wall basic replaced by fibrous tissue, muscle tissue infarction area and the infarction area boundary, and myocardial infarction area basic cell death, replaced by fibroblasts and collagen tissue, the ligation of coronary artery has definite myocardial infarction and ventricular wall tissue reconstruction. At the same time, the cardiac function of the model group was dramatically decreased, and the serum CK-MB and LDH activities were dramatically increased. In summary, all the results confirmed that the model of AMI was successful.

Apoptosis is a form of programmed cell death that occurs in an organism. It is a characteristic change and death of a cell caused by a biochemical event. These changes include cell shrinkage, nuclear rupture, chromatin condensation, and chromosomal DNA fragmentation [21]. In the process of MI, mitochondrial dysfunction is one of the main mechanisms leading to myocardial cell damage [22]. During myocardium ischemia, calcium overload in myocardial cells will lead to increased calcium content in the mitochondria, which leads to mitochondrial swelling and membrane communication. Then, myocardial cell permeability changes, metabolic pressure increases, and the process of myocardial cell necrosis and apoptosis begins with the increase of mitochondrial membrane permeability [23]. The NDRG is a family of new genes that have been gradually discovered in recent years. The role of family members in oncology has been studied by many researchers [24]. However, recent studies have pointed out that NDRG family genes also play a crucial role in the heart. Researcher indicates that NDRG4 is specifically expressed in the heart tissues [25] and that NDRG4 is indispensable for the development of zebrafish heart [26]. At the same time, we detected the expression of NDRG family genes in rat heart tissues and found that NDRG4 expression was most dramatically inhibited. From this, we speculated that NDRG4 can protect myocardial cell damage caused by MI.

Next, we used transfection technology to overexpress NDRG4 in H9C2 cells, and the H9C2 cells were treated with I/H. First, Elisa results showed that overexpression of NDRG4 could effectively protect H9C2 cells and reduce the activity of CK-MB and LDH. The activity of CK-MB and LDH is often used to measure the damage degree of myocardial cells. When the cells are stimulated, CK-MB and LDH secreted by the cells will enter the extracellular fluid through the damaged cell membrane. At the same time, overexpression of NDRG4 can reverse I/H-induced decrease in H9C2 cell viability. In the process of cardiomyocyte apoptosis, the Bcl-2 family is a regulator that plays a very important role in it [27]. It is mainly divided into two categories according to function, including proapoptotic proteins Bax and Bnip-3 and antiapoptotic proteins Bcl-2 and Bcl-XL. These factors can interact to jointly regulate the apoptosis of cardiomyocytes [11]. Among them, Bcl-2 and Bcl-XL are the most important antiapoptotic factor, and Bax is the most important proapoptotic factor, which plays a crucial role in the regulation of apoptosis [28]. With the increase of Bcl-2 protein expression, more and more Bax dimers are separated from each other to form a more stable Bax-Bcl-2 heterodimer, thus neutralizing the apoptotic effect of Bax dimer. That is, the ratio of Bax/Bcl-2 determines the survival and death of cells. When the expression of Bcl-2 protein exceeds Bax protein, it can inhibit apoptosis, and when the expression of Bax protein exceeds Bcl-2 protein, it can promote apoptosis. A large number of studies have confirmed that after culturing H9C2 cells in an I/H environment, Bax dimers increased dramatically and there appeared cell apoptosis. In our study, after H9C2 cells overexpressed NDRG4, the Bax/Bcl-2 ratio was dramatically reduced; also, the protein expression of Bcl-XL was dramatically increased. And TUNEL staining confirmed that the apoptosis rate of H9C2 cells was reduced after overexpression of NDRG4. This suggested that NDRG4 has a significant role in inhibiting H9C2 cell apoptosis. In order to further verify the protective effect of NDRG4 in the heart, we injected Ad in the left ventricle of the rat to overexpress NDRG4, and through echocardiography and hemodynamic detection of the corresponding indicators, it was found that heart tissue of rats after overexpression of NDRG4 can dramatically improve the heart function reduction caused by MI, and rat serum LDH and CK-MB activity was also dramatically reduced. H&E staining further confirmed that NDRG4 can improve cardiac structure. These results further confirmed the protective effect of NDRG4 on the heart.

The JAK/STAT pathway is a crucial intracellular signal transduction pathway that has received much attention in recent years and is involved in a variety of physiological processes that mediate cell growth, proliferation, differentiation, and apoptosis [29]. Studies have pointed out that the JAK/STAT pathway is activated during I/R injury, thereby regulating the biological activity of downstream substrate molecules through phosphorylation [30]. However, the current view is that the effect of the JAK/STAT pathway on myocardial tissue is unclear. At the same time, some studies have pointed out that the JAK/STAT pathway can regulate cardiomyocyte apoptosis by regulating the expression of Bcl-2 and Bax [31]. In this study, we found that the JAK2/SATA3 pathway was activated in H9C2 cells induced by I/H treatment, while NDRG4 can effectively inhibit the phosphorylation levels of JAK2 and SATA3, thereby inhibiting the expression of downstream apoptotic genes.

## 5. Conclusion

The expression of NDRG4 is downregulated in myocardial infarction tissue, while overexpression of NDRG4 in cardiac tissue can dramatically improve cardiac structure and function. At the same time, overexpression of NDRG4 in H9C2 cells can effectively inhibit the I/H-induced decrease in cell viability and increase in apoptosis rate, and it may be through the inhibition of the JAK2/STAT3 signaling pathway.

## Figures and Tables

**Figure 1:** Changes of cardiac function and structure after MI in rats. (a–j) Echocardiography and hemodynamic testing in rats. (k, l) Elisa was used to detect the LDH and CK-MB content in serum. (m) H&E staining was used to detect the change of cardiac structure, bar = 25 *μ*M (“∗” indicates statistical difference from the Sham group, *P* < 0.05).

**Figure 2:** MI induces myocardial cell apoptosis and downregulation of NDRG expression. (a) Immunohistochemical staining was used to detect the expression of Caspase3 and semiquantitative analysis, bar = 25 *μ*M. (b) Western blot was used to detect the expression of Bax, Bcl-2 and Bcl-XL in heart tissues and protein band analysis. (c, d) qRT-PCR was used to detect the expression of Bax, Bcl-2, Bcl-XL, NDRG1, NDRG2, NDRG3, and NDRG4 in heart tissues (“∗” indicates statistical difference from the Sham group, *P* < 0.05).

**Figure 3:** Overexpression of NDRG4 can inhibit H9C2 cell apoptosis induced by I/H. (a) qRT-PCR was used to detect the expression of NDRG4 in H9C2 cells. (b) CCK-8 assay was used to detect the cell viability. (c, d) Elisa was used to detect the LDH and CK-MB content in cell supernatant. (e) TUNEL staining was used to detect the apoptosis level in H9C2 cells and positive rate analysis, bar = 50 *μ*M. (f) Western blot was used to detect the expression of Bax, Bcl-XL, and Bcl-2 in H9C2 cells and protein band analysis. (g) qRT-PCR was used to detect the expression of Bax, Bcl-XL, and Bcl-2 in H9C2 cells (“∗” indicates statistical difference from the Normoxia group, *P* < 0.05; “#” indicates statistical difference from the I/H+OE-NC group, *P* < 0.05).

**Figure 4:** Overexpression of NDRG4 in rat heart can improve MI-induced cardiac function and structural damage. (a) qRT-PCR was used to detect the expression of NDRG4 in heart tissues. (b–k) Echocardiography and hemodynamic testing in rats. (l, m) Elisa was used to detect the LDH and CK-MB content in serum. (n) H&E staining was used to detect the change of cardiac structure, bar = 25 *μ*M (“∗” indicates statistical difference from the MI group, *P* < 0.05; “#” indicates statistical difference from the MI+Ad-NC group, *P* < 0.05).

**Figure 5:** NDRG4 inhibits the activation of the JAK2/STAT3 pathway induced by I/H. (a) Western blot was used to detect the expression of p-JAK2, JAK2, p-STAT3, and STAT3 in H9C2 cells and protein band analysis. (b) The ratio analysis of p-JAK2/JAK2 and p-STAT3/STAT3 (“∗” indicates statistical difference from the Normoxia group, *P* < 0.05; “#” indicates statistical difference from the I/H+OE-NC group, *P* < 0.05).

## Data Availability

The data used to support the findings of this study are available from the corresponding author upon request.

## Supplementary Materials

Supplementary 1 Supplementary Table 1: antibody information.

Supplementary 2 Supplementary Table 2: real-time PCR primers.
